RETRACTED

# Gender Identification and Classification of *Drosophila melanogaster* Flies Using Machine Learning Techniques

**DOI:** 10.1155/2022/4593330

**Published:** 2022-01-13

**Authors:** Channabasava Chola, J. V. Bibal Benifa, D. S. Guru, Abdullah Y. Muaad, J. Hanumanthappa, Mugahed A. Al-antari, Hussain AlSalman, Abdu H. Gumaei

**Affiliations:** ^1^Department of Computer Science and Engineering, Indian Institute of Information Technology, Kottayam, India; ^2^Department of Studies in Computer Science, University of Mysore, Karnataka, India; ^3^Sana'a Community College, Sana'a 5695, Yemen; ^4^Department of Computer Science and Engineering, College of Software, Kyung Hee University, Suwon-si 17104, Republic of Korea; ^5^Department of Computer Science, College of Computer and Information Sciences, King Saud University, Riyadh 11543, Saudi Arabia; ^6^Computer Science Department, Faculty of Applied Sciences, Taiz University, Taiz 6803, Yemen

## Abstract

*Drosophila melanogaster* is an important genetic model organism used extensively in medical and biological studies. About 61% of known human genes have a recognizable match with the genetic code of Drosophila flies, and 50% of fly protein sequences have mammalian analogues. Recently, several investigations have been conducted in Drosophila to study the functions of specific genes exist in the central nervous system, heart, liver, and kidney. The outcomes of the research in Drosophila are also used as a unique tool to study human-related diseases. This article presents a novel automated system to classify the gender of Drosophila flies obtained through microscopic images (ventral view). The proposed system takes an image as input and converts it into grayscale illustration to extract the texture features from the image. Then, machine learning (ML) classifiers such as support vector machines (SVM), Naive Bayes (NB), and *K*-nearest neighbour (KNN) are used to classify the Drosophila as male or female. The proposed model is evaluated using the real microscopic image dataset, and the results show that the accuracy of the KNN is 90%, which is higher than the accuracy of the SVM classifier.

## 1. Introduction

Drosophila fly is considered as one of the most effective organisms for analysing the root causes of human diseases. The Drosophila is used for medical research because of the fact that their internal organ systems functions similar to those in vertebrates, including humans. Few differences exist between humans and Drosophila in terms of their cellular features and gross morphological; however, many of biological, physiological, and neurological properties are conserved between both the organisms. It should be necessary to mention that about 75% of human disease-related genes are believed to have functional similarity in the fly [1]. Neurological and developmental disorders, cardiovascular disease, cancer, and metabolic and storage diseases, as well as genes required for the auditory and function of the visual and immune systems are also matching with the genes of Drosophila [2]. Several assays have been developed in the recent years on drosophila, and they are used for the investigation of human diseases. These include nervous system assays such as hearing, learning, memory, and diurnal rhythmicity which have been conducted in Drosophila, and the outcomes are used to study the neurological dysfunction, including epilepsy, neurodegeneration, dementias, stroke, brain tumours, and traumatic brain injury [3]. *Drosophila melanogaster* is used as a model organism to study Alzheimer's disease, and it is further related to decline in cognitive function, social withdrawal, poor judgement, and short-term memory loss [4]. Despite the fact that the fruit fly Drosophila has never been utilized in asthma research, it could be incredibly useful in tying genetic processes to biological utilities [5].

RETRACTED

*Drosophila melanogaster* male and female can be differentiated by their size of the body as shown in Figure 1. The size of the body is associated with genotype and phenotype of the flies that indirectly affects the size of flies and the gender classification process. Handa et al. (2014) stated that the size of flies operates in an opposite direction for the two genders because of the presence of polymorphism in Drosophila [6].

The polymorphism size is one of challenging tasks in the gender classification process. Gender identification of drosophila fruit flies is important for biologists to study the aging effects, Alzheimer disease, neural degenerative illness, and medical assays before performing any experimentation. Because the sizes of drosophila flies are very small in nature and difficult to classify by inexpert humans, there is an urgent need to use image processing with machine learning methods for gender identification of drosophila fruit flies and speeding up the experiments on them. Moreover, the gender discrimination of drosophila can help to understand the behavioural patterns in the natural life environment [6].

Different approaches have been proposed to classify the gender of *Drosophila melanogaster* based on the wings of the fly. Ahmad et al. (2014) proposed an approach to extract wing texture features (both sign and magnitude) of male and female using local binary patterns and modified local binary patterns along with SVM and random forest (RF) classification algorithms [7]. The approach employed the texture feature to divide the images into regions of interest and then classify those regions. Moreover, the texture feature also offers information in the spatial procedure of colours or intensities in the input image [7]. The authors achieved 84% average accuracy for the gender classification through wing texture feature extraction. Neto et al. (2017) proposed the gender classification based on wings with the help of stationary wavelet transformation, canny filter, and fractal dimension as features and applied SVM and RF classifiers for classification tasks [8]. For shape retrieval, the histogram of oriented gradients (HOG) features and KNN classifier are used to categorize the class based on spatial relationship [9]. It is also a well-known fact that only limited research has been carried out till date in the area of *Drosophila* gender classification through computational methods. Further, none of the related works addressed the Drosophila gender classification using ventral view datasets.

RETRACTED

In this proposed work, we propose a machine learning-based intelligent approach to classify and identify the gender of *Drosophila melanogaster* from microscopic images (ventral view) for developing one of the intelligent systems in e-health and medical services.

The remainder of the article is organized as follows. In Section 2, the high level work flow of the proposed method is presented. In Section 3, experimental results and discussion on comparative analysis are summarized, followed by the concluding remarks in Section 4.

## 2. Proposed Methodology

Image classification is one of the most prominent parts of image processing domain. The high-level work flow of proposed methodology to identify and classify the Drosophila gender from microscopic image datasets is presented in Figure 2. The proposed method includes four stages, namely, dataset collection, preprocessing, feature extraction, and classification.

### 2.1. Dataset Collection

Standard Drosophila image dataset is not available publicly; hence, the Drosophila images were captured in the National Drosophila Stock Centre, Department of Studies in Zoology, University of Mysore, India, with a digital compound microscope. The microscopic image dataset contains 100 images with two different classes, namely, male and female in which each class of 50 images are collected. These Drosophila images are captured at different lighting conditions which pose the challenges such as variation in viewpoint, illumination and background. Images of live flies are captured by anaesthetizing then placing it on the stages of microscope at perfect view point. The sample images of male and female Drosophila flies are displayed in Figure 3 where the upper row consists of female, and the lower row with male flies.

RETRACTED

### 2.2. Preprocessing

Preprocessing is performed to enhance the quality and appearance of the training and test images. The colour images are converted into binary images by setting a threshold value to perform the segmentation process in the image. The RGB input image is of size *m* × *n* × 3, and these images are resized to *m* × *n* size before converted into grayscale. In the proposed methodology, the colour images (RGB format) are resized to 256 × 256 and converted into grayscale images for extracting the gray level cooccurrence features. Subsequently, the preprocessed images are passed for extracting useful features.

### 2.3. Feature Extraction

Feature extraction is the process of extracting the high-level information from an image such as colour, shape, and texture. In the proposed work, texture features are considered for classifying the *Drosophila melanogaster*. Statistical techniques are employed to study the spatial distribution of gray values by computing the local features at each point in an image. The gray level cooccurrence matrix (GLCM) and texture feature extraction strategies are introduced by Haralick et al. in 1973 [10, 11]. Haralick feature extraction technique is widely used in image analysis applications, and it is a two-step process as shown in Figure 4. The GLCM consists of computed texture features based on each pixel's grey level value, which is located at or related to fixed geometric position [10]. The texture descriptors given in Equations (1) to (17) are used in the present work. Here, (*i*, *j*) defines the (*i*, *j*)^th^ element of the normalized GLCM highlighted in Figure 4 [12]. Here, contrast is a measure of gray level variations or intensity between the seed pixel and the neighbourhood pixels where higher contrast reflects higher intensity variations in GLCM.

The expression used for measuring the contrast is presented in Equation (1), where *p*_*d*_ is the probabilities calculated for pixel values in GLCM.

(1) $$\begin{array}{c} \text{contrast}=\underset{k}{\sum }\underset{l}{\sum }{\left(k-l\right)}^{2}P_{d}\left(k,l\right). \end{array}$$

Homogeneity is used to measure the closeness and distribution of elements in the diagonal pixel of GLCM. As the homogeneity becomes higher, it tends to reduce the contrast. The expression for measuring the homogeneity is given in

(2) $$\begin{array}{c} \text{homogeneity}=\underset{\text{k}}{\sum }\underset{\text{l}}{\sum }\frac{1}{1+{\left(\text{k}‐\text{l}\right)}^{2}}\;p_{d}\left(k,l\right). \end{array}$$

Entropy feature is a measure of randomness or a degree of disorderliness existed in the image. It employs the principal statistical features to estimate the variations between pixel intensities. The expression for measuring entropy is presented in Equation (3).

(3) $$\begin{array}{c} \text{Entropy}=\underset{k}{\sum }\underset{l}{\sum }\frac{1}{1+{\left(k-l\right)}^{2}}\;\ln\;p_{d}\left(k,l\right). \end{array}$$

$\text{Energy}=\sqrt{\beta }$ can be obtained from the angular second moment (*β*), where the *β* value gives the gray level local uniformity of. It is essential to note that the higher similarity leads to larger *β* value. Considering the energy value, the expression used to compute *β* is presented in

(4) $$\begin{array}{c} \beta =\underset{k}{\sum }\underset{l}{\sum }{p_{d}}^{2}\left(k,l\right). \end{array}$$

Correlation feature is known as the linear dependency of gray level values in the cooccurrence matrix, and it is given in

(5) $$\begin{array}{c} \text{Correlation}=\underset{k}{\sum }\underset{l}{\sum }p_{d}\left(k,l\right)\frac{\left(k-\mu_{x}\right)\left(l-\mu_{y}\right)}{\sigma_{x}\sigma_{y}}, \end{array}$$

where *μ*_x_, *μ*_*y*_ and *σ*_x_, *σ*_*y*_ are the means and standard deviations in *x* and *y* directions, respectively, and are expressed in

(6) $$\begin{array}{c} \mu_{x}=\underset{k}{\sum }\underset{l}{\sum }{kp}_{d}\left(k,l\right), \end{array}$$

(7) $$\begin{array}{c} \mu_{y}=\underset{k}{\sum }\underset{l}{\sum }{lp}_{d}\left(k,l\right), \end{array}$$

(8) $$\begin{array}{c} \sigma_{x}=\sqrt{\underset{k}{\sum }\underset{l}{\sum }{\left(k-\mu_{x}\right)}^{2}p_{d}\left(k,l\right)}, \end{array}$$

(9) $$\begin{array}{c} \sigma_{y}=\sqrt{\underset{k}{\sum }\underset{l}{\sum }{\left(l-\mu_{y}\right)}^{2}p_{d}\left(k,l\right)}. \end{array}$$

The moments can be defined as statistical expectation of a random variable for certain power functions. It is categorised by the following: moment 1 (*m*_1_) is the average or the mean of pixels values within an image, and it is written in Equation (10). Moment 2 (*m*_2_) represents the standard deviation, which is expressed in Equation (11). Moment 3 (*m*_3_) defines the degree of asymmetry in the distribution as expressed in Equation (12). Finally, moment 4 (*m*_4_) feature gives the flatness of a distribution or relative-peak, and it is also termed as kurtosis as given in Equation (13).

(10) $$\begin{array}{c} m_{1}=\underset{k}{\sum }\underset{l}{\sum }\left(k-l\right)P_{d}\left(k,l\right), \end{array}$$

(11) $$\begin{array}{c} m_{2}=\underset{k}{\sum }\underset{l}{\sum }{\left(k-l\right)}^{2}P_{d}\left(k,l\right), \end{array}$$

(12) $$\begin{array}{c} m_{3}=\underset{k}{\sum }\underset{l}{\sum }{\left(k-l\right)}^{3}P_{d}\left(k,l\right), \end{array}$$

(13) $$\begin{array}{c} m_{4}=\underset{k}{\sum }\underset{l}{\sum }{\left(k-l\right)}^{4}P_{d}\left(k,l\right). \end{array}$$

Furthermore, different statistics that are known to be a subset of the cooccurrence matrix are also used in the present mathematical model. The statistical features depend on the probability distribution *P*_*x*−*y*_(*z*), which is defined in Equation (14).

(14) $$\begin{array}{c} P_{x-y}\left(z\right)=\underset{k}{\sum }\underset{l}{\sum }C_{d}\left(k,l\right),z=0,1,.\cdots \cdots ,N_{g}-1, \end{array}$$

where *N*_*g*_ is the number of gray levels in the normalized symmetric GLCM of dimension *N*_*g*_ × *N*_*g*_, *C*_*d*_(*k*, *l*) is the (*k*, *l*)^th^ element of the GLCM. The simple different statistic descriptions of textures are the angular second moment, mean, and entropy which are expressed in Equations (15), (16), and (17), respectively.

(15) $$\begin{array}{c} \beta =\sum {\left(P_{x-y}\left(z\right)\right)}^{2}. \end{array}$$

If the *P*_*x*−*y*_(*z*) values are close or very similar, then *β* attains the small value. Alternatively, *β* be large when certain values of *P*_*x*−*y*_(*z*) increases and remaining magnitudes are low.

(16) $$\begin{array}{c} \text{Mean}=\underset{z}{\sum }{zP}_{x-y}\left(z\right). \end{array}$$

When the values of *P*_*x*−*y*_(*z*) are focused on near the origin, the obtained mean value is less, and mean is large when they are located far from the origin.

(17) $$\begin{array}{c} \text{Entropy}=-\underset{z}{\sum }P_{x-y}\left(z\right)\;\log\;P_{x-y}\left(z\right). \end{array}$$

Entropy reaches minimum value when *P*_*x*−*y*_(*z*) values are unequal, and it reaches the high magnitudes while *P*_*x*−*y*_(*m*) values are equal. Haralick's texture feature extraction using the above equations is applied for the preprocessed image database of Drosophila. Gray level cooccurrence texture features such as contrast, entropy, homogeneity, correlation, energy, mean, *m*_1_, *m*_2_, *m*_3_, *m*_4_, and *β* exist for all images.

RETRACTED

### 2.4. Classification

In the proposed work, the ventral views of *Drosophila melanogaster* obtained from microscopic colour images (50 male and 50 female) are considered as the dataset. Classification is a labelling task of the data into specific predefined classes based on the knowledge base of the features [20]. In the present work, SVM [13], KNN [14], and NB [15] classification algorithms are employed, and the appropriate explanations are added in Section 2.4 (i), (ii), and (iii), respectively.

- Support vector machines

The SVM is a widely used machine learning (ML) method based on statistical learning theory [16, 17]. SVM is employed for classification of images and information in multiple domains because of its higher accuracy. SVM is subsample learning method that works on the principle of structural risk minimization. It works on pattern recognition problem and builds hyperplanes in high-dimensional space for classification [19]. Optimal hyperplanes are constructed by iterative training process that subsequently reduces the error in classification. The standard SVM is used for binary classifier problems that learns by differentiating two classes with maximum margin and generates support vectors.

Let us consider a training set of labelled instances that are pair linear functions expressed as (*M*_*i*_, *F*_*i*_), *i* = 1, 2, ..⋯*N* where *M*_*i*_ ∈ {1,−1}^*N*^. The SVM classifier classifies the data using Equation (18).

(18) $$\begin{array}{c} f\left(x\right)=W^{T}X+b, \end{array}$$

where *X* is the training samples, *W* is the weights assigned, and *b* is bias or offset.

(ii) Naive Bayes classifier

The NB is a simple probabilistic classifier works based on generic statement that all features are independent category variables. NB classifier works based on the Bayes theorem as expressed in Equation (19), which considers the assumption of naive (strong) independence. NB classifier assumes that the effect of a value for a variable on a given class is independent of the value of another variable. This assumption is termed class conditional independence. NB can be utilized for more sophisticated classification problems especially, when the dimensionality of the inputs is high. When more competent output is needed, as compared to other classification methods, NB implementation can be used. Moreover, NB is also used to create models with predictive capabilities. On the other hand, Bernoulli distributions or discrete feature multinomials are widely used [15].

(19) $$\begin{array}{c} P\left(A\;|\;\;B\right)=\frac{P\left(B\;|\;A\right).P\left(A\right)}{P\left(B\right)}, \end{array}$$

*P*(*B* | *A*):Probability of *B* being true given that A is true.

P(A |  *B*):Probability of A being true given that *B* is true.

*P*(*B*):Probability of *B* being true.

*P*(*A*):Probability of A being true.

(iii) *K*-nearest neighbour classifier

KNN is a simple classification algorithm works on the principle of selection of *k*-nearest data points to classify into appropriate classes. It uses the distance measures to compare the similarity between two classes [14]. The KNN operates on the principle that related samples fitting to the same class have high probability. Initially, *K* value has to be selected for each sample followed by the prediction of test samples [18]. In the present work, Euclidean distance is employed between training and testing vector, and it is given in Equation (20). In Equation (20), dist(*e*, *f*) specifies the Euclidean distance between points *e* and *f*.

(20) $$\begin{array}{c} \text{dist}\left(e,f\right)=\sqrt{\overset{n}{\underset{i=1}{\sum }}{\left(e_{i}-f_{i}\right)}^{2}}. \end{array}$$

The label of shortest distance feature vector is considered to be the testing vector.

RETRACTED

### 2.5. Evaluation Metrics

The performance of the proposed method is evaluated in terms of accuracy, precision, recall, and *F*-score as explained subsequently.

- Precision: it is the fraction of retrieved items that are relevant for the classification results

(21) $$\begin{array}{c} \text{Precision}=\frac{\#\left(\text{relevant items retrieved}\right)}{\#\left(\text{retrieved items}\right)}. \end{array}$$

(ii) Recall: it is related to information retrieval and can be defined as the fraction of the items successfully retrieved that are relevant to the query

(22) $$\begin{array}{c} \text{Recall}=\frac{\#\left(\text{relevant items retrieved}\right)}{\#\left(\text{relevant items}\right)}. \end{array}$$

(iii) *F*-score: it is a measure of tests' precision and recall and can be computed by their values and scores. The balanced *F*-score or traditional *F*-score (also called *F*-measure) is considered a harmonic mean for both recall and precision

The performance of the system is computed in terms of its accuracy, *F*-score, precision, and recall as given in

(23) $$\begin{array}{c} \text{Accuracy}=\frac{\left(\text{TP}+\text{TN}\right)}{N}, \end{array}$$

(24) $$\begin{array}{c} \text{Precision}=\frac{\text{TP}}{\left(\text{TP}+\text{FP}\right)}, \end{array}$$

(25) $$\begin{array}{c} \text{Recall}=\frac{\text{TP}}{\left(\text{TP}+\text{TN}\right)}, \end{array}$$

(26) $$\begin{array}{c} \text{F}1‐\text{Score}=2\times \left(\frac{\left(\text{Precision}\times \text{Recall}\right)}{\left(\text{Precision}+\text{Recall}\right)}\right), \end{array}$$

where TP is true positive, TN is true negative, FP is false positive, and FN is false negative for the overall test samples *N*.

## 3. Experimental Results and Discussion

The proposed research work is implemented using MATLAB 2019 (a) installed in a computing machine with i7 processor with 32 GB RAM. The results corresponding to the Drosophila gender identification using various classifiers are analyzed in this section. For the experimentation, a unique dataset is created, and the ventral views of Drosophila images are considered for preprocessing. The preprocessed images are fed to feature extraction, and the extracted features are given to the supervised classifiers. Supervised classification methods need training samples with labelled data to do the classification task [21]. The efficiency of proposed classification algorithm is calculated using precision, recall, *F*-measure, and accuracy [22].

RETRACTED

The accuracy of various classifiers with respect to Haralick's features is presented in Figure 5. For experimentation, initially, the *K*-value is set as 1, 5, 10, 20, and the squared root of sample size is assumed, and the finest results are conveyed. In NB classifier, *α* is fixed to 1, and *β* is tuned for Bernoulli and multinomial event models. When the training samples are 90% and test samples are 10%, KNN achieves the maximum accuracy about 90%. Subsequently, SVM achieves a classifier accuracy of 80%, and NB has the least accuracy of 40%. It is evident that when the number of training samples is increased KNN performs effectively because of its nearest neighbourhood property.

Next, consider the case of 70% images for training and 30% for testing. In this case, SVM has the accuracy of 73.33% followed by KNN achieving 70%, and NB attains 60% accuracy. When the number of training samples is reduced, the performance of KNN and SVM classifiers are decreased while the performance of NB is improved. It is observed that when the number of images in the training samples is more, then KNN can be utilized for classification purpose. Further, SVM can be used when 60-70% samples are used for training, and NB is employed when the number of training images is kept in minimum.

The *F*-measure results obtained for SVM, KNN, and NB classifiers with different training-testing sample percentage are presented in Figure 6. The results prove that KNN achieves highest test accuracy for different cases. For training-testing percentage such as (90%, 10%) and (50%, 50%), it achieves a test accuracy of 88% and 66.66%. Considering SVM, for 90% testing and 10% training samples, it achieves a test accuracy of 83%. It also achieves a test accuracy of 48.78% for 50% training and 50% test samples. NB achieves an *F*-measure about 40% for the case with 90% training and 10% testing samples. Subsequently, *F*-measure about 61.81% is achieved for 50% training and 50% test images by NB classifier. In summary, KNN is efficient while compared to other classifiers in terms of the *F*-measure analysis for Drosophila dataset followed by SVM and NB.

The precision analysis of Drosophila dataset in terms various classifiers are presented in Figure 7. Precision analysis is done for various classifiers with Drosophila dataset, and the results indicate KNN, SVM, and NB achieve a precision of 100%, 71.42%, and 40%, respectively, in terms of 90% training and 10% test images. When the number of images in training dataset is reduced, and the number test images is increased, then various changes are observed in the results. For 80% training and 20% testing images, KNN, SVM, and NB achieves a precision of 100%, 72.2%, and 57.14%, respectively. Subsequently, when the number of training and testing images is 70% and 30%, respectively, there is a drastic change in the precision factor of KNN such that the precision is 75%. When the number of images is further reduced in the training set, the precision factor of KNN is slightly improved. However, considering the overall results, KNN offers a good average precision about 87%. Alternatively, while considering the case of SVM classifier, it achieves an average precision of 69.9%. The NB is also analysed for precision factor, and it attains an average precision of 53.76%. Therefore, it is evident that KNN achieves the maximum precision while compared with the other classification methods.

RETRACTED

The recall analysis of various classifiers in terms of the given Drosophila dataset is presented in Figure 8. From the recall analysis, it is evident that the KNN, SVM, and NB classifiers achieve a recall factor of 80%, 100%, and 40%, respectively, in terms of 90% training and 10% test images. When the number of images in training samples is reduced and the test images are increased, significant changes are observed in the results. For the case of 80% training and 20% testing images, KNN, SVM, and NB achieve a recall of 70%, 80%, and 40%, respectively. Subsequently, when the number of training and testing images is changed into 70% and 30%, respectively, recall factor of KNN also reduced to the value of 60%. However, considering the overall results, SVM achieves an average recall factor of 67.74%, and NB classifier achieves an average recall of 52.6%. The KNN is also analysed for recall factor, and it attains an average recall of 64.2%. So, it is evident that SVM achieves the maximum recall factor while compared with the other methods.

KNN exhibits amazing performance in such a way that it almost achieves the minimal error rate as compared with Bayes optimization under trivial conditions. The performance of KNN method is affected by multiple constraints, such as the selection of the *K*-value and the selection of distance measures. KNN is sensitive to *K*-values and selects *K*-closest training samples from the Drosophila dataset. The running cost of KNN is also minimal while compared to SVM and NB classifiers. The running cost of KNN, SVM, and NB classifiers while operated on Drosophila dataset with 50 and 90 samples are given in Figures 9 and 10, respectively. KNN has achieved minimum running cost in seconds while compared to SVM and NB classifiers. NB shows poor performance because of increased computational operations while compared with other techniques.

RETRACTED

SVM is a popular method that proves to be robust and offers global optimal solutions for Drosophila gender classification problem. The complexity factor of SVM relies on the support vectors (SV) apart from input space dimension. Subsequently, the SV extracted from the Drosophila dataset have data complexity that varies when the SVM is applied for other classification problems. The SV captured for Drosophila dataset has an upper bound (half the size of training samples) based on the class separability and data dimensions. Instances with dissimilar labels distribute the input space to stop a linear hyperplane from accurate classification. In the input space, the learning process of a nonlinear boundary rises some computational requirements during the optimization phase. The optimization phase in SVM learns only a linear discriminant surface in the mapped space during Drosophila gender classification.

For reducing the error and cost factor while training the Drosophila dataset, SVM executes supplementary constraint such as the hyperplane needs to be positioned at an extreme distance from various classes. This process facilitates the optimization step to determine the generalized hyperplane that are mandatory. It is a well-known fact that testing and training can be done on dissimilar samples, so the test samples may have unrelated distributions than the subsamples trained on. This leads to the reduction of accuracy of the classifiers and it also affects the other metrics.

## 4. Conclusion

In the presented work, a model to identify the gender of *Drosophila melanogaster* based on microscopic images (ventral view) is demonstrated. The model uses Haralick's method for texture feature extraction, and the extracted features are given to the classifier. The proposed model employs SVM, KNN, and NB for doing the classification task. This method offered efficient results in detecting the gender of the Drosophila flies. The proposed method is evaluated with the Drosophila dataset collected from Mysore University, India, and shows good accuracy in classification. The presented novel Drosophila gender classification method is evaluated in terms of accuracy, recall, precision, and *F*-measure scores. In the comparison analysis of SVM, KNN, and NB, the accuracy of KNN is 10% higher than SVM, and the computational cost of KNN is comparatively lower than the SVM, and the accuracy result achieved by this work is 90%. This outcome can be applied to different medical research activities for identifying the gender of the Drosophila flies and utilizing in various diagnostic and genetic researches. In future work, we plan to collect a large size dataset and various views, also video-based near real time analysis gender of drosophila, and should consider improvement in aspect performance and robustness with deep learning-based techniques for classification of gender and various task-related *Drosophila melanogaster* flies.

RETRACTED

## Figures and Tables

**Figure 1:** Enlarged microscopic images of Drosophila flies.

**Figure 2:** High-Level work flow of proposed methodology.

**Figure 3:** Example photographs of Drosophila under a microscope.

**Figure 4:** Haralick texture features computation.

**Figure 5:** Classifiers accuracy analysis for Drosophila dataset.

**Figure 6:** Classifiers *F*-measure analysis for Drosophila dataset.

**Figure 7:** Classifiers precision analysis for Drosophila dataset.

**Figure 8:** Classifiers recall analysis for Drosophila dataset.

**Figure 9:** Running cost of various classifiers for Drosophila dataset with 50 samples.

**Figure 10:** Running cost of various classifiers for Drosophila dataset with 90 samples.

## Data Availability

The data used to support the findings of this study are available from the corresponding author upon request.
